The article "Cardioprotective properties of N-terminal galanin fragment (2-15) in experimental ischemia/reperfusion injury" was published in 2017. Journal: Oncotarget.

# Cardioprotective properties of N-terminal galanin fragment (2-15) in experimental ischemia/reperfusion injury

**DOI:** 10.18632/oncotarget.21503

**Published:** 2017-10-05

**Authors:** Oleg Pisarenko, Andrei Timotin, Maria Sidorova, Irina Studneva, Valentin Shulzhenko, Marina Palkeeva, Larisa Serebryakova, Aleksander Molokoedov, Oksana Veselova, Mathieu Cinato, Frederic Boal, Helene Tronchere, Oksana Kunduzova

**Affiliations:** ^1^ Russian Cardiology Research and Production Complex, Moscow, Russian Federation; ^2^ National Institute of Health and Medical Research (INSERM) U1048, Toulouse, France; ^3^ University of Toulouse, UPS, Institute of Metabolic and Cardiovascular Diseases, Toulouse, France

**Keywords:** galanin (2-15), apoptosis, cardiac injury, energy metabolism, oxidative stress

## Abstract

**Background and purpose:**

Galanin is an endogenous peptide involved in diverse physiological functions in the central nervous system including central cardiovascular regulation. The present study was designed to evaluate the potential effects of the short N-terminal galanin fragment 2-15 (G) on cardiac ischemia/reperfusion (I/R) injury.

**Experimental Approach:**

Peptide G was synthesized by the automatic solid phase method and identified by 1H-NMR spectroscopy and mass spectrometry. Experiments were performed on cultured rat cardiomyoblast (H9C2) cells, isolated perfused working rat hearts and anaesthetized open-chest rats.

**Key Results:**

Cell viability increased significantly after treatment with 10 and 50 nM of G peptide. In hypoxia and reoxygenation conditions, exposure of H9C2 cells to G peptide decreased cell apoptosis and mitochondrial reactive oxygen species (ROS) production. Postischemic infusion of G peptide reduced cell membrane damage and improved functional recovery in isolated hearts during reperfusion. These effects were accompanied by enhanced restoration of myocardial metabolic state. Treatment with G peptide at the onset of reperfusion induced minor changes in hemodynamic variables but significantly reduced infarct size and plasma levels of necrosis markers.

**Conclusion and implications:**

These findings suggest that G peptide is effective in mitigating cardiac I/R injury, thereby providing a rationale for promising tool for the treatment of cardiovascular diseases.

## INTRODUCTION

Galanin, a 29/30 amino acid neuropeptide, is widely distributed throughout the central and peripheral nervous system as well as endocrine system, preferentially in brain, hypothalamus, pituitary, and other tissues including the heart. Galaninergic system is involved in multiple regulatory functions, including central cardiovascular control [1]. The N-terminal fragments of galanin are crucial for its biological activity and the first 15 amino acids are conserved in most species [2], while the C-terminal region (residues 17-29) varies among species and lacks receptor affinity [2]. To date, three galanin receptors (GalR1, GalR2 and GalR3), members of the GPCR superfamily, have been identified by molecular cloning and pharmacologically characterized [3].

The article "Cardioprotective properties of N-terminal galanin fragment (2-15) in experimental ischemia/reperfusion injury" was published in 2017. Journal: Oncotarget.

GalR1 and GalR3 activate the intracellular effectors through pertussis toxin (PTX) sensitive Gi/o proteins, which results in the inhibition of adenylyl cyclase activity and a decrease in cAMP in the cytosol that leads to the opening of G protein gated inwardly-rectifying potassium (GIRK) channels [4, 5]. Additionally, GalR1 activation stimulates MAPK activity in a PKC-independent manner by coupling with a G_i_-type G-protein via Gβγ subunits [6]. GalR2 triggers PLC activity via Gα_q/11_-proteins, leading to IP3-mediated opening of Ca^2+^-dependent channels and release of Ca^2+^ into the cytoplasm from intracellular stores [7]. GalR2 is also able to activate MAPK through PKC and Gα_o_-proteins dependent mechanism leading to the downstream PI3K-dependent phosphorylation of Akt resulting in suppression of caspase-3 and caspase-9 activity [8]. GalR2 activation also inhibits forskolin stimulated cAMP production in a PTX-sensitive manner, suggesting the activation of Gα_i/_α_o_-proteins [8]. Thus, activation of all galanin receptors can inhibit the formation of the transcription factor cAMP regulatory element binding protein (CREB) [8]. Noteworthy, the activated CREB may inhibit the Rab GTPase-activating protein (AS160), a substrate of Akt and glucose transporter 4 (GLUT4) translocation, thus promoting insulin resistance [9]. The differences in the functional coupling and subsequent signaling activities contribute to the diversity of galanin physiological effects. Although the galanin signaling has been characterized in neuronal cells, carcinoma cells and rat gastrointestinal tract [10], the role of GalR-mediated signaling pathways in the heart is poorly explored.

The cardiovascular effects of galanin and its fragments are complex. These peptides are involved in central cardiovascular control affecting arterial pressure and heart rate (HR). Administration of galanin into the rostral ventrolateral medulla produced a hypotensive effect by reducing the sympathetic vasomotor tone in rats [10]. Intracisternal injections of galanin or its fragments (1–15) and (1–16) produce a transient vasopressor response followed by a decrease in mean arterial pressure (MAP) which is accompanied by tachycardia in rats [10]. It has been demonstrated that cardiovascular action of galanin occurs by interactions of its receptors with α_2_-adrenergic receptors and angiotensin II receptor type 1 and neuropeptide Y1 receptor subtypes [1]. Infusion of human galanin into male volunteers increased resting HR by decreasing vagal tone and stimulated the release of growth hormone (GH) [11], thus indicating that this peptide is able to modulate GH secretion and vagal control of the heart. Galanin may have a direct action on cardiomyocytes, since all three galanin receptor subtypes are expressed in the heart [5, 12]. However, the available data on the effects of galanin peptides on cardiac function are scanty. In isolated guinea pig papillary muscle galanin exerted a positive inotropic action and prolonged effective refractory period [13]. These effects may be associated with galanin-induced activation of inwardly rectifying K^+^ channels, in cardiac myocytes [14]. Under hypoxic conditions, galanin may protect the cardiac muscle against contractile disturbances through activation of ATP-sensitive K^+^ channels [13, 14]. The ability of galanin to gate ATP-sensitive K^+^ channels and hyperpolarize membrane potential was also demonstrated in the insulinoma cell line RINm5F [15]. Galanin mRNA levels in cardiac sympathetic neurons and myocardial galanin content are increased one week after cardiac ischemia and reperfusion in rats [16]. The increase in galanin content specifically in the damaged left ventricle is consistent with studies showing that the peptide is transported to regenerating nerve endings after axon damage [16, 17]. In addition, galanin stimulates sensory nerve regeneration and may promote the re-growth of cardiac sensory nerves following ischemia-reperfusion [18, 19]. These observations suggest that galaninergic system plays an important role in the pathophysiology of many diseases at the level of central cardiovascular regulation. However, the peripheral function of galanin and its fragments remains to be determined.

The article "Cardioprotective properties of N-terminal galanin fragment (2-15) in experimental ischemia/reperfusion injury" was published in 2017. Journal: Oncotarget.

Therefore, we aimed to investigate the effects of G peptide on *in vitro* in H9C2 cardiomyoblast cell line subjected to hypoxia/reoxygenation (H/R), *ex vivo* in isolated perfused rat hearts and *in vivo* in a rat model of I/R injury.

## RESULTS

### The effects of G on H9C2 cell survival in response to stress

To determine whether G affects cell viability, we examined the dose-dependent effects of the peptide on H_2_O_2_-induced loss of ATP in H9C2 cells. As shown in Figure 1, cell exposure to 400 μM H_2_O_2_ for 4 hours led to a significant reduction of the cell viability compared to control. Dose-response studies revealed that G at the dose of 10 and 50 nM was able to prevent H_2_O_2_-induced decrease of ATP levels. Next, we examined by TUNEL assay whether G affects apoptotic cell death in response to hypoxic stress. Because 50 nM of G produced approximately a 20 % increase in cardiomyoblast viability, we used this concentration in subsequent experiments. As shown in Figure 2, the exposure of H9C2 cells to hypoxia caused an increase in the number of TUNEL-positive cells as compared to normoxia. However, the treatment of cells with 50 nM G significantly reduced hypoxia-induced apoptosis (Figure 2).

**Figure 1:** Dose-dependent effect of G on cell viability in response to oxidative stress Treatment of cardiomyoblasts with G prevents H_2_O_2_-induced decrease of cell viability in a dose-dependent manner. The H9C2 were pretreated with G (10, 50, 250 nM) for 20 min and then exposed to 400μM H_2_O_2_ for 4h. Values are the means ± SEM for three experiments. ^*^P < 0.05 vs H_2_O_2_ treatment; ^**^P < 0.01 vs H_2_O_2_ treatment; ^§§§^*P* < 0.001, vs control.

**Figure 2:** Effect of G on hypoxia-induced cell apoptosis **(A)** Representative fluorescence images of H9C2 cells pretreated with 50 nM G for 20 min and then exposed to normoxia or hypoxia-reoxygenation. Apoptosis was measured by TUNEL assay in H9C2 cells after 16h of hypoxia followed by 3h of reoxygenation. **(B)** Quantitative analysis of TUNEL-positive cells in H9C2 cells. The arrows indicate apoptotic cells. Values are the means ± SEM from three experiments. ^***^P < 0.001, vs normoxia (C); ^§§§^*P* < 0.001, vs hypoxia (H).

### The effects of G on hypoxia-induced mitochondrial ROS production in H9C2 cells

The excessive generation of ROS and impaired cellular metabolism are closely linked to cell death and myocardial damage [20]. To determine whether G could affect ROS generation, we examined the effects of G on mitochondrial superoxide (O_2_^-^) production using the MitoSOX Red fluorescent probe. As shown in Figure 3A, 3B, cell exposure to hypoxic stress caused a significant increase in O_2_^-^ production as compared to normoxia. Importantly, treatment of H9C2 cells with 50 nM G markedly prevented hypoxia-induced O_2_^-^ formation (Figure 3).

**Figure 3:** Effect of G on hypoxia-induced mitochondrial O_2_^-^ production **(A)** Representative fluorescence images of H9C2 cells pretreated with G peptide. Mitochondrial O_2_^-^ formation was assessed by MitoSOX RED in H9C2 cells exposed to 16h hypoxia followed by 3h of reoxygenation. **(B)** Quantitative analysis of O_2_^-^ production in H9C2 cells exposed to normoxia or hypoxia-reoxygenation. Values are the means ± SEM from three experiments. ^*^P < 0.05 vs normoxia; ^##^*P* < 0.01 vs hypoxia.

### Effects of exogenous G in isolated rat heart subjected to I/R injury

Infusion of peptide G after global ischemia enhanced recovery of cardiac function during reperfusion compared with control. A concentration-dependent effect of G on recovery of CO at the end of reperfusion is shown on Figure 4A. The maximal response to G infusion was observed at the concentration of 225 μM; at higher peptide concentrations CO recovery reduced. А similar effects were obtained for recovery of the index of contractile function intensity expressed as LVDP×HR product (Figure 4B). Comparison of the main cardiac function indices for 225 μM G infusion and control is shown in Table 1. In addition to enhanced recovery of CO and LVDPxHR product, the recovery of LV systolic pressure, aortic output and stroke volume was also significantly higher whereas LV diastolic pressure and coronary resistance were markedly reduced in the G group compared with these indices in control. Thus, administration of the optimal concentration of peptide G at the onset of reperfusion caused a pronounced reduction of I/R injury.

The article "Cardioprotective properties of N-terminal galanin fragment (2-15) in experimental ischemia/reperfusion injury" was published in 2017. Journal: Oncotarget.

**Figure 4:** Effects of peptide G concentrations in KHB on recovery of cardiac output **(A)** and the index of contractile function intensity **(B)** at the end of reperfusion. Values are means ± SEM from 8 experiments and are expressed in percentage of the initial value. CO, cardiac output; LVDP×HR, the index of contractile function intensity. The dotted lines show recovery of the indices in control.

**Table 1:** Effect of infusion of 225 μM G after global ischemia on recovery of isolated rat heats at the end of reperfusion

	Steady state	Control	G
Coronary flow, ml/min	17 ± 2	13 ± 1^a^	15 ± 1
Perfusion pressure, mmHg	62 ± 3	58 ± 1	61 ± 1
Coronary resistance, mmHg/ml	3.65 ±0.03	4.46 ±0.07^a^	4.06 ±0.10^ab^
LV systolic pressure, mmHg	98 ± 3	69 ± 1^a^	85 ± 2^ab^
LV diastolic pressure, mmHg	-3 ± 1	10 ± 1^a^	5± 1^ab^
LV developed pressure, mm Hg	101± 1	59 ± 2^a^	80 ± 3^ab^
Heart rate, beat/min	302 ± 2	240 ± 3^a^	245 ± 3^a^
LVDP x HR, mmHg/min	30380 ±373	14186 ±525^a^	19474 ± 643^ab^
Aortic output, ml/min	26 ± 3	0 ± 1^a^	12 ± 1^ab^
Cardiac output, ml	43 ± 2	13 ± 1^a^	27 ± 2^ab^
Stroke volume, μl	142 ± 1	54 ± 4^a^	110 ± 4^ab^

The hearts were perfused as indicated in Materials and methods. Data are the mean ± SEM for 8 experiments. ^a^ P<0.05 vs. steady state;^b^ P<0.05 vs. control.

We evaluated the effects of 225 μM G infusion on the energy state of reperfused hearts and LDH leakage during early reperfusion. The hearts of the control group exhibited a poor restoration of high-energy phosphates, significant decrease in the total creatine (ΣCr) and lactate accumulation in myocardial tissue at the end of reperfusion compared with the steady state (Figure 5). Postischemic G infusion significantly enhanced restoration of ATP, ΣAN and increased adenylate energy charge (AEC) in reperfused hearts compared with control. These effects were combined with a significant increase in PCr recovery, better preservation of ΣCr and a substantial reduction in myocardial lactate content. LDH leakage in the perfusate before ischemia did not differ significantly between the studied groups (Figure 6A). In control, the release of LDH at early reperfusion increased by more than two-fold compared with the value before ischemia. G infusion significantly decreased LDH leakage compared with control, thus suggesting fewer defects of the sarcolemma. *In vivo* studies on activity of necrosis marker showed that plasma level of CK-MB and LDH increased by 8 and 20 times respectively, at the end of reperfusion in the control animals (Figure 6B, 6C). Administration of G at dose of 0.35 or 2.10 μmol/kg did not significantly reduce the activity of both enzymes compared with control. However, treatment with G at dose of 0.7 or 1.4 μmol/kg reduced the CK-MB and LDH activity (on average 1.6 and 1.5-times respectively, compared to the values in the control group). Decrease in the plasma activity of both necrosis markers in the group G-1.4 is shown in Figure 6B, 6C. These experiments demonstrated a direct cardioprotective action of exogenous peptide G on the heart after ischemia and reperfusion.

The article "Cardioprotective properties of N-terminal galanin fragment (2-15) in experimental ischemia/reperfusion injury" was published in 2017. Journal: Oncotarget.

**Figure 5:** Effect of G infusion on energy state of isolated rat heart at the end of reperfusion St. st. - steady state; G - 5-min infusion of 225 μ M G after ischemia. **(A)** Myocardial contents of ATP and ΣAN=ATP+ADP+AMP. **(B)** Adenylate energy charge (AEC) = (ATP+0.5ADP)/ΣAN. **(C)** Myocardial contents of PCr and total creatine ΣCr=PCr+Cr. **(D)** Myocardial content of lactate. Values are the means ± SEM from 8 experiments. ^*^P < 0.05 vs. steady state; ^#^P < 0.05 vs. control.

**Figure 6:** Effects of G administration on necrosis markers in *ex vivo* and *in vivo* models of myocardial I/R injury **(A)** LDH release in myocardial effluent from isolated perfused rat heart. Control - postischemic infusion of KHB; G - postischemic infusion of KHB with 225 μM G. Values are the means ± SEM of 8 experiments and are expressed in IU/g dry wt. for 5-min Langendorff perfusion before or after global ischemia (early reperfusion). ^*^ p<0.05 vs. the value before ischemia; ^#^ p<0.05 vs. the value in control. Activities of LDH **(B)** and CK-MB **(C)** in blood plasma in rats *in vivo*. St. state - steady state; Control – i.v. administration of saline at the onset of reperfusion; G - i.v. administration of peptide G (1.4 μmol/kg) at the onset of reperfusion. Values are the means ± SEM for 8 experiments.^*^ P<0.05 vs. steady state; ^#^ P<0.05 vs. control.

The article "Cardioprotective properties of N-terminal galanin fragment (2-15) in experimental ischemia/reperfusion injury" was published in 2017. Journal: Oncotarget.

### Effects of G administration in rats with myocardial regional ischemia and reperfusion

Changes in hemodynamic variables in rats treated with increasing doses of peptide G are shown in Table 2. Mean systolic arterial pressure (SAP) and heart rate (HR) did not differ significantly between studied groups in the steady state. Bolus injection of saline after the period of LAD coronary artery occlusion did not affect SAP and HR during reperfusion in control. Postischemic administration of any dose of peptide G resulted in a transient rise in SAP followed by its decrease (on average by 10±1 and 26±3% of the initial value at the first minutes of reperfusion). By the end of reperfusion, SAP recovered to near baseline (94±3%). A decrease in HR was observed in all G-treated groups at the first minute of reperfusion (on average by 10±1% from baseline). Further reperfusion resulted in HR restoration in the groups G-0.35 and G-2.10. In the other two groups, HR decreased on average by 18±2% of the steady state value. By the end of reperfusion, HR did not differ from baseline values in all G-treated groups.

**Table 2:** Effects of i.v. G administration on hemodynamic variables in anesthetized rats *in vivo*

Group	Steady state	LAD reperfusion		
		1-2 min	2-3 min	60 min
SAP, mm Hg				
Control	90 ± 4	88 ± 2	87 ± 2	86 ± 3
G-0.35	86 ± 2	97 ± 3^ab^	73 ± 2^ab^	82 ± 4
G-0.70	87 ± 2	94 ± 2^ab^	71 ± 2^ab^	80 ± 2
G-1.40	89 ± 3	97 ± 3^b^	76 ± 3^ab^	85 ± 2
G-2.10	85 ± 3	94 ± 3	72 ± 3^ab^	81 ± 3
HR, beats /min				
Control	321 ± 12	315 ± 8	313 ± 8	308 ± 5
G-0.35	312 ± 11	290 ± 7	308 ± 7	296 ± 7
G-0.70	328 ± 9	295 ± 10^a^	287 ± 9^ab^	302 ± 6
G-1.40	314 ± 10	274 ± 7^ab^	261 ± 7^ab^	292 ± 6
G-2.10	319 ±12	297 ± 8	328 ± 9	299 ± 9

Peptide G was administrated by i.v. bolus injection at the onset of reperfusion at doses of 0.35, 0.70, 1.40 or 2.10 μmol/kg (groups G-0.35, G-0.70, G-1.40 or G-2.10, respect.). An equal volume of saline was injected in control. Values are expressed as mean ± SEM for 8 experiments. Significant difference (P<0.05) from: ^a^ steady state; ^b^ control.

The percentage ratios of AAR/LV did not differ significantly in all studied groups. AAR/LV in the control group and the mean AAR/LV value in G-treated groups were 39.6±0.7 and 40.8±1.0%, respect. Peptide G administration at a dose of 0.35 μmol/kg did not affect the percentage ratio of MI/AAR compared with control (40.8±1.3 and 40.7±2.1%, respectively) (Figure 7). Administration of the peptide at dose of 0.7 and 1.4 μmol/kg significantly reduced the percentage ratio of MI/AAR (on average by 22±1% compared with the value in control), thus indicating limitation of infarct size. Infarct size did not significantly differ from control in the group G-2.10.

The article "Cardioprotective properties of N-terminal galanin fragment (2-15) in experimental ischemia/reperfusion injury" was published in 2017. Journal: Oncotarget.

**Figure 7:** Effects of intravenous G administration on myocardial infarct size (MI/AAR, %,) in rats *in vivo* Black circle corresponds to myocardial infarction in control. Values are means ± SEM from 8 experiments.^*^P < 0.05 vs. control.

The results of *in vivo* study showed that i.v. administration of peptide G slightly affected systemic hemodynamic parameters but significantly reduced irreversible myocardial damage induced by LAD coronary artery occlusion followed by reperfusion.

## DISCUSSION

Galanin is involved in regulating numerous of pathological and physiological processes, through interactions with three G-protein-coupled receptors, GalR1-3. Over the past decade, it was shown that both agonists and antagonists for galanin receptor subtypes can be used as putative therapeutics targets for the treatment of various human diseases. These compounds exhibit an antidepressant and anxiolytic efficacy in animal models, have adhesive and antidepressant properties and may be also useful as potential regulators of feeding behavior and agents for the treatment of Alzheimer's disease [21]. In addition to the complete peptide, several truncated galanin fragments are also biologically active [12]. In the current study, we provide the first *in vitro*, *ex vivo* and *in vivo* evidence that short galanin fragment G reduces I/R-induced injury in the heart. Using live-cell model we show that G prevents mitochondrial ROS production in response to stress. Several lines of evidence suggest that excessive ROS generation in mitochondria may provoke a state of oxidative stress, associated with pathophysiological progression in heart ischemic diseases [22]. In addition, in cardiomyoblasts exposed to hypoxia, G is able to reduce apoptotic cardiac cell death suggesting that G may control activation of apoptotic cell death pathways and oxidative stress during stressful conditions. These effects may be related to an increase in enzymatic antioxidant capacity induced by the peptide or the antioxidant action. Indeed, we have previously demonstrated that some endogenous peptides such as apelin, may exhibit powerful antioxidant properties [23, 24]. Signaling via GalR1-3 receptors triggers multiple intracellular routes that mimic postconditioning. Unfortunately, the non-selectivity of galanin (2-15) to GalR1-3 receptors excludes more specific suggestions. Undoubtedly, reduction in mitochondrial ROS formation may be one of the operative mechanisms contributing to less cell damage. In addition, galanin-induced cardioprotection is associated with a reduction in infarct size after acute reperfusion. This finding implies the activation of survival kinase pathways that prevents opening of the mPTP. But the functional involvement of these mechanisms can be confirmed only by using inhibitors of signaling cascades and antioxidants. Exploration of the nature of cardioprotective properties of galanin deserves further expanded research.

The article "Cardioprotective properties of N-terminal galanin fragment (2-15) in experimental ischemia/reperfusion injury" was published in 2017. Journal: Oncotarget.

A short-term postischemic G infusion caused the concentration-dependent recovery of cardiac function during reperfusion of isolated rat heart. Noteworthy, the optimal peptide concentration effectively restored metabolic state of reperfused heart and reduced cell membrane damage. Intravenous injection of G at the onset of reperfusion also exerted the dose-dependent limitation of myocardial infarct size in rats along with the concomitant decrease in activity of necrosis markers in blood plasma. These data suggest, for the first time, that peptide G may act as postconditioning agent effectively reducing reperfusion injury.

Galaninergic system plays an important role in determining the status of cardiovascular system in pathological states. Our findings identify G peptide as a potent protective agent in mitigating metabolic disturbance in the heart. Importantly, the preservation of metabolic status of the myocardium after I/R stress was associated with reduction in infarct size and improvement of cardiac function. Our previous study has demonstrated that galanin fragment (2-11) has a role in regulating biological activity of cardiac cells under stress conditions [20]. At the same time, it is not possible to evaluate the contribution of GalR1, GalR2 and GalR3 receptors to G effects based on the obtained results. Indeed, several of the physiological effects modulated by galanin may be mediated via both GalR2 and GalR3 subtypes activation. GalR2 couples to PLC mediated via G_q/11_ and hence activates the MAPK pathways (ERK) and Akt leading to inhibition of caspase-3 and caspase-9, thus reducing apoptotic cell death [4, 6, 8, 20, 25]. Additionally, PLC activation increases inositol phosphate hydrolysis, mediating the release of Ca^2+^ into the cytoplasm from intracellular stores and opening Ca^2+-^dependent chloride channels [4, 7, 20]. Signaling via GalR3 coupled to a Gi/o-type G-protein stimulates PTX-sensitive opening of GIRK channels [4, 5, 26]. Lastly, GalR2 and GalR3 activation inhibits the phosphorylation of CREB [4, 6, 27], which leads to GLUT4 translocation from intracellular membrane compartments to plasma membranes to enhance glucose uptake [28, 29]. All these mechanisms are implicated in recovery of cardiac function and reduction of irreversible cardiomyocyte damage in the heart subjected to I/R injury. Therefore, further studies are required to identify the precise role of these receptors in cardioprotective activity of G peptide.

The article "Cardioprotective properties of N-terminal galanin fragment (2-15) in experimental ischemia/reperfusion injury" was published in 2017. Journal: Oncotarget.

The involvement of galaninergic signaling in a variety of physiological and pathological functions amplify interest in investigation of agonist and antagonists of GalR1-3 receptors for the correction of cardiac disturbances in ischemic heart disease and heart failure. Recently it was shown that the GalR1 antagonist M40 attenuated remodeling and improved cardiac function in a rat model of HF [30]. The beneficial effects of M40 are attributed to suppression of the inhibitory action on the vagal nerve induced by galanin in HF and improvement of the balance of the autonomic nervous system and cardiac function. These data suggest that GalR1 antagonist may be a potential therapeutic agent for HF. On the other hand, our recent studies demonstrate that galanin fragment (2-11) can enhance metabolic and functional tolerance to I/R stress [20]. Although the deletion of the Gly^1^ residue results in loss of affinity for GalR1 [31], further delineation of cardioprotective mechanisms against I/R injury requires the development of selective agonists.

In conclusion, by combining *in vitro*, *ex vivo* and *in vivo* approaches, we show that G peptide is effective in mitigating myocardial I/R injury. These data provide the first evidence that G treatment after ischemia improved recovery of cardiac function and reduced infarct size. The preservation of cardiac function by the G was accompanied by restoration of myocardial energy state and cell membrane integrity. In addition, G attenuates mitochondrial ROS production and apoptosis in cardiomyoblasts in response to hypoxic stress. Taken together, these results indicate that peptide G may be a promising tool for the treatment of myocardial I/R damage.

## MATERIALS AND METHODS

### Galanin (2-15)

Galanin fragment (2-15) H-Trp-Thr-Leu-Asn-Ser-Ala-Gly-Tyr-Leu-Leu-Gly-Pro-His-Ala-OH (G) was synthesized by solid-phase method on a Tribute-UV peptide synthesizer (Protein Technologies Inc., USA) according to standard protocol for condensation of Fmoc-amino acids using *O-*(benzotriazole-1-yl)-1,1,3,3,-tetramethyluronium tetrafluoroborate (TBTU). Amino acid side chain functional groups were blocked with the acid labile protecting groups: tert-butoxycarbonyl (Boc) at indole moiety of Trp; tert-butyl (But) at hydroxyl groups of Ser, Thr and Tyr; trityl (Trt) at imidazole ring of His; and at carboxamide function of Asn. Fmoc-Ala-Wang resin (capacity 0.64 mmol/g) was used as the starting material. All amino acids were coupled as active derivatives in a 4-fold excess with the use of the TBTU with addition of N-methylmorpholine coupling method. Cleavage of the Fmoc group was carried out with 25% 4-methylpiperidine in *N,N*-dimethylformamide. After synthesis had been completed, side chain deprotection and cleavage of peptide from a solid support were performed by treatment with a solution containing 90% TFA, 2.5% water, 5% dithiothreitol and 2.5% triisobutylsilane for 1.5 h at 20 °C. The peptide was precipitated with dry diethyl ether. Crude peptide was purified by HPLC. Preparative HPLC was performed on a Knauer (Germany) system using Eurosphere C18 column (20 × 250mm, 10 μm particle size) (Knauer, Germany). The elution was achieved with a linear gradient of acetonitrile (B) in aqueous 0.1% TFA (A) at a flow rate of 10 ml/min with UV detection at 220 nm. Purity of the peptide (96.6%) was checked by an analytical HPLC with Luna 100 C18 (2) column (4.6×250 mm, 5 μm particle size) with linear gradient of acetonitrile in aqueous 0.1% TFA. Peptide structure was confirmed by both ^1^H-NMR and mass spectrometry techniques. ^1^H-NMR spectra were obtained using a WM-500 spectrometer (Bruker, Germany). Mass-spectrometry data were obtained using an Ultrafex MALDI TOF/TOF (Bruker Daltonics, Germany) instrument.

The article "Cardioprotective properties of N-terminal galanin fragment (2-15) in experimental ischemia/reperfusion injury" was published in 2017. Journal: Oncotarget.

### Reagents

Fmoc-protected amino acids derivatives were purchased from Novabiochem and Bachem (Switzerland). Chemicals for peptide synthesis were from Fluka (Switzerland). Enzymes and chemicals were purchased from Sigma Chemical Co. (St Louis, MO USA). Solutions were prepared using deionized water (Millipore Corp. Bedford, MA, USA).

### Animals

Male Wistar rats weighing 300 to 340 g were housed in cages in groups of three, maintained at 20–30°C with a natural light-dark cycle. All animals had free access to standard pelleted diet (Aller Petfood, St. Petersburg, Russia) and tap water. They were purchased in the Pushchino Nursery for laboratory animals, Russian Academy of Sciences. The care and use of the animals were conducted in accordance with the European Convention for the Protection of Vertebrate Animals Used for Experimental and other Scientific Purposes (No 123 of 18 March 1986).

### Isolated perfused rat hearts

Rats were heparinized by intraperitoneal injection (1600 IU/kg body weight) and anaesthetized with urethane (i.p., 1.3 g/kg body weight). Hearts were perfused with Krebs-Henseleit buffer (KHB) supplied with 11 mM glucose. A needle was inserted into the left ventricular (LV) cavity to register LV pressure via a Gould Statham P50 transducer, SP 1405 monitor and a Gould Brush SP 2010 recorder (Gould, Oxnard, Ca, USA). The contractile function intensity index was calculated as the LV developed pressure-heart rate product (LVDP×HR), where LVDP is the difference between LV systolic and LV end-diastolic pressure. Cardiac pump function was assessed by cardiac output (CO), the sum of aortic output and coronary flow [20].

The article "Cardioprotective properties of N-terminal galanin fragment (2-15) in experimental ischemia/reperfusion injury" was published in 2017. Journal: Oncotarget.

The steady state values of cardiac function were recorded after preliminary 20-min perfusion in working mode according to a modified method of Neely under constant left atrium pressure and aortic pressure of 20 and 100 cm H_2_O, respectively. After the steady state period, the control hearts were perfused with KHB in Langendorff mode for 5 min at a constant flow rate of 4 ml/min, and then they were subjected to 35-min normothermic global ischemia followed by 5-min Langendorff reperfusion in the same mode with subsequent 25-min working reperfusion by Neely method. In the G group, 5-min Langendorff reperfusion at a constant flow rate of 4 ml/min with KHB containing 75, 150, 175, 225, 275 or 290 μM G was applied after global ischemia. Other experimental stages were the same as in control. After preliminary working perfusion (steady state) and at the end of reperfusion, the hearts were freeze-clamped in liquid nitrogen for metabolite analysis. The myocardial effluent was collected in ice-cold tubes during both periods of Langendorff perfusion for assessment of LDH activity.

### Analysis of metabolites

Frozen tissue of the left ventricle (LV) of the heart was quickly homogenized in cooled 6% HClO_4_ (10 ml/g) using an Ultra-Turrax T-25 homogenizer (IKA-Labortechnik, Staufen, Germany), and the homogenates were centrifuged at 2800×g for 10 min at 4°C. The supernatants were then neutralized with 5 M K_2_CO_3_ to pH 7.40, and the extracts were centrifuged after cooling to remove KClO_4_ precipitate. Tissue dry weights were determined by weighing a portion of the pellets after extraction with 6% HClO_4_ and drying overnight at 110°C. Concentrations of ATP, ADP, AMP, phosphocreatine (PCr), creatine (Cr) and lactate in neutralized tissue extracts were determined by enzymatic methods [20].

### Anesthetized rats *in vivo*

Rats were anesthetized with 20% urethane (120 mg/kg body wt i.p.) and artificially ventilated with a KTR-5 animal respirator (Hugo Sacks Electronik) with a volume of 2–3 ml at a rate of 70–75 breaths/min. Further preparation of animals was performed as described earlier [27]. Arterial blood pressure was recorded with a pressure transducer (Statham p23Db, Oxnard, USA) using a polygraph Biograph-4 (St. Petersburg, Russia). The mean arterial pressure, HR and standard lead II ECG were recorded on a computer using a LabVIEW 7.1 data acquisition system (National Instruments, USA) [20].

The article "Cardioprotective properties of N-terminal galanin fragment (2-15) in experimental ischemia/reperfusion injury" was published in 2017. Journal: Oncotarget.

In control, after 30-min stabilization of hemodynamic parameters (steady state), LAD coronary artery was occluded for 40 min to simulate regional ischemia; the duration of subsequent reperfusion was 1 h. Prior to intravenous administration, G was dissolved in saline. In the experimental series, G was administrated by i.v. bolus injection at the onset of reperfusion at doses of 0.35, 0.70, 1.40 and 2.1 μmol/kg (groups G-0.35, G-0.7, G-1.4 and G-2.1, respect.) An equal volume of saline (0.5 ml) was injected in control. At the end of experiments, LAD coronary artery was reoccluded and 2 ml of 2% Evans Blue (Sigma, USA) solution was injected through the jugular vein to distinguish the myocardial non-ischemic area from the area at risk (AAR).

### Determination of myocardial infarct size

After staining with Evans Blue, the heart was excised and the LV was frozen. A frozen LV was transversely cut into 1.5 mm thick slices which were incubated in 0.1 M sodium phosphate buffer pH 7.40, containing 1% 2,3,5-triphenyl-tetrazolium chloride (TTC, Sigma, USA) 10 min at 37°C. The slices were fixed in 10% formalin for 5 min. Then they were placed between two transparent glasses and captured on both sides using a scanner at 600 d.p.i. resolution; the saved images were analyzed by computerized planimetry using Imagecal software. The slices were then weighed for determination of LV weight. The AAR was expressed as a percentage of LV weight, myocardial infarction (MI) was expressed as a percentage of the AAR in each group [20].

### Determination of necrosis markers

At the end of the steady state and reperfusion, blood samples were collected for plasma separation. Plasma LDH activity was determined enzymatically with pyruvate as substrate by using standard kits from BioSystems S.A. (Barcelona, Spain). Plasma CK-MB activity was assessed by an immunoinhibition method using standard kits from BioSystems S.A. (Barcelona, Spain) from the rate of NADPH formation in the hexokinase and glucose-6-phosphate dehydrogenase coupled reactions.

### Cell culture and treatments

Rat ventricular myocardial H9C2 cells were obtained from American Type Culture Collection (Manassas, VA, USA). H9C2 cells at passages 18 to 24 were seeded in 24 or 96-well cell culture plates with Dulbecco's Modified Eagle Medium (Invitrogen, Cergy-Pontoise, France) containing 10% Fetal Bovine Serum (Invitrogen, Cergy Pontoise, France), 100U mL^-1^ penicillin and 100μg mL^-1^ streptomycin at 37°C in a humidified atmosphere of 5% CO_2_ and were used at less than 80% of confluence.

### Measurement of mitochondrial O_2_^-^ production

The mitochondrial levels of ROS were determined in H9C2 cells subjected to hypoxia (1% O_2_, 5% CO_2_, 94% N2) for 16h followed by 4h of reoxygenation (95% O_2_, 5% CO_2_) using mitochondrial superoxide indicator (MitoSOX^TM^ red, Life Technologies). Before hypoxia the H9C2 were pretreated with G for 20 min. After reoxygenation, cells were washed once with PBS and incubated in 1μM MitoSOX red for 30 min at 37°C followed by three washes with PBS. The fluorescence was then measured at the excitation wavelength of 510 nM and emission wavelength of 580 nM.

The article "Cardioprotective properties of N-terminal galanin fragment (2-15) in experimental ischemia/reperfusion injury" was published in 2017. Journal: Oncotarget.

### Evaluation of apoptosis

The apoptosis level was assessed using the TUNEL system according to manufacturer's instructions (Promega, Madison, WI, USA) as described previously [22]. TUNEL is a general method to detect nuclear DNA fragmentation during apoptosis. TUNEL technique relies on the use of endogenous enzymes that allow the incorporation of labeled nucleotides into the 3′-hydroxyl (3′OH) recessed termini of DNA breaks. The added value in this approach resides in the possibility of evaluating both morphological and staining features in the same sample.

### ATP measurement

ATP was measured with the CellTiter-Glo^®^ Luminescent Cell Viability Assay from Promega (Madison, WI). H9C2 cells were seeded at a density of 2 × 10^5^ cells/ml with 100 μl per well in a white 96-well plate and allowed to grow for 24 h. Before addition of 400 μM of H_2_O_2_ for 4 h, H9C2 cells were pretreated for 20 min with G at the different doses (10, 50 and 250 nM). The cells were equilibrated at room temperature for 30 min and, followed by addition of the CellTiter-Glo^®^ reagents, per manufactured instructions. The luminescence was read after a 10 min incubation of the reagents on the INFINITE F500 on luminescence module (TECAN, Switzerland, Mennedorf) and expressed as mean percentage of control group.

### Statistical analysis

Data are presented as means ± SEM. Results were analyzed by one-way ANOVA followed by Bonferroni multiple range test post-hoc analysis for calculation differences between more than two groups. Comparisons between two groups involved use of the Student's unpaired t-test. All statistical analyses were performed using SigmaPlot version 12 (Systat Software Inc, San Jose, CA). P < 0.05 was defined as significant. The data and statistical analysis complied with the recommendations on experimental design and analysis in pharmacology [23].

### Nomenclature of targets and ligands

Key protein targets and ligands in this article are hyperlinked to corresponding entries in http://www.guidetopharmacology.org, the common portal for data from the IUPHAR/BPS.

## Abbreviations

AAR: area at risk
AEC: adenylate energy charge
Boc: tert-butoxycarbonyl
BUT: tert-butyl
CK-MB: creatine kinase-MB
CO: cardiac output
ΣCr: total creatine
Cr: creatine
CREB: cAMP responsive element
G: galanin fragment (2-15)
GAL: galanin
GalR: galanin receptor (1, 2, 3)
GH: growth hormone
GIRK: gated inwardly-rectifying potassium
GLUT4: glucose transporter 4
^1^H-NMR: proton nuclear magnetic resonance
HF: heart failure
H/R: hypoxia/reoxygenation
HR: heart rate
I/R: ischemia/reperfusion
KHB: Krebs-Henseleit buffer
LAD: left anterior descending artery
LV: left ventricular
LVDP: left ventricular developed pressure
MAP: mean arterial pressure
MI: myocardial infarction
PCr: phosphocreatine
PTX: pertuxis toxin
SAP: systolic arterial pressure
TBTU: *O-*(benzotriazole-1-yl)-1,1,3,3,-tetramethyluronium tetrafluoroborate
TFA: trifluoroacetic acid
TTC: 2,3,5-triphenyl-tetrazolium chloride
